# Cyclic Fatigue Resistance of Nickel–Titanium Rotary Instruments after Simulated Clinical Use

**DOI:** 10.1155/2022/1716008

**Published:** 2022-10-11

**Authors:** Hana R. Ubaed, Diyar Kh. Bakr

**Affiliations:** Conservative Department, Hawler Medical University, Erbil 44000, Iraq

## Abstract

**Objective:**

Cyclic fatigue occurred in the curved canal when the instrument freely rotated leading to repeated compressive and tensile stresses. This study aims to evaluate the cyclic fatigue resistance (CFR) of new and used 2Shape and AF F-One rotary instrument systems by using an artificial stainless-steel canal.

**Methods:**

A total of 80 rotary nickel–titanium (NiTi) instruments of two systems were used, 2Shape/TS2 and AF F-ONE/F5 (40 in each group). The instruments were subdivided into group A 20 instruments (10 per system) that remain unused, group B 20 instruments (10 per system) instrumented 20 root canals (each file prepared 1 canal for 2 minutes), group C 20 instruments (10 per system) instrumented 40 canals each for 2 minutes (each file prepared 2 canals), group D of 20 instruments (10 per system) prepared 60 canals each for 2 minutes (each file prepared 3 canals). After each canal instrumentation, the instruments were cleaned and sterilized by autoclave. Then, all the instruments underwent cyclic fatigue testing in an artificial stainless steel canal with a 50° canal curvature and a radius of curvature of 5 mm. The time and number of cycles to failure (NCF) were recorded. Data were analyzed using the Welch ANOVA test for intragroup comparison and the pairwise test for multiple comparisons.

**Results:**

The unused instruments of the AF F-One rotary system showed statistically higher CFR than clinically used instruments (*P* < 0.05). 2Shape system was not affected by clinical use (*P* > 0.05). The mean NCF of AF F-One instruments was significantly higher than the equivalent file group of 2Shape instruments (*P* < 0.05).

**Conclusion:**

A reduction in the CFR for AF F-One instruments after use was observed when compared to the new unused file group. The 2Shape system was not affected by clinical use. AF F-One performed better in terms of NCF.

## 1. Introduction

Nickel–titanium (NiTi) rotary instruments have assisted dentists in debriding and root canal preparation; despite this clear advantage, they still have some risk of the fracture without any visible sign [1, 2].

Failure of instruments used in rotational motion occurs in two ways: torsional fatigue and flexural fatigue. Torsional failure occurs when the tip of the instrument is locked in the canal while the shank continues to rotate [3], and in the second scenario, cyclic/flexural fatigue happens by repeated tensile and compressive loads when the instrument rotates freely in a curved canal and does not bind until a fracture occurs [4, 5].

An instrument fracture may be influenced by numerous factors such as the technique of preparation, rotational speed, manufacturing technology, radius of canal curvature, and angle of canal curvature. Furthermore, the authors found that clinical use, exposure to sodium hypochlorite (NaOCl), and autoclave sterilization procedures affected the mechanical properties of NiTi instruments, thereby decreasing the cyclic fatigue resistance (CFR) of these instruments [6–8].

Manufacturers have developed several strategies to overcome these problems, including a modification in instrument design, create new NiTi alloys, and use new activation kinematics [9, 10]. Moreover, manufacturers developed several manufacturing methods such as ion implantation, electro-polishing, heat treatment, and thermo-mechanical techniques to enhance the resistance to cyclic fatigue [10–12].

The 2Shape (Micro-Mega, France) instrument is a new group of the endodontic file system that uses T-wire technology to enhance the CFR of endodontic instruments by 40% and the flexibility of the files [13].

AF F-One (Fanta Dental Material Co., Shanghai, China) is a rotary NiTi instrument that was developed and specified by a flat-sided S-shaped cross-section, and it is used in continuous rotation motion with an inactive tip and 25/0.06 taper. The design of this instrument offers advantages of increasing fatigue lives and reducing blade engagement [14].

The CFR significantly decreased by the repeated use of NiTi instruments [15], although there is no agreement on the exact number of uses allowed before the instrument fails. Studies presented that cyclic fatigue is the main cause of instrument fracture and surface deformation occurred on the files because of clinical usage [16]. As there are limited studies comparing the CFR of 2Shape and AF F-One rotating NiTi instruments before and after clinical use, the aim of this study was to evaluate the CFR of TS2/2Shape and AF F-One/Fanta in dissimilar situations before and after clinical use as follows; new unused instruments, and instruments tested after the clinical preparation of one, two, or three mandibular premolars with one straight root canal, by analyzing the time and number of cycles required to fracture the instruments.

## 2. Materials and Methods

80 rotary NiTi instruments (length = 25 mm) from two systems (20 per system) were used in this study, as follows: 2Shape/TS2 (tip 25, taper 0.06) and AF/F-One (tip 25, 0.06 taper). Before performing the cyclic fatigue tests, the instruments were inspected under a stereomicroscope (Motic ST-39 Series, China) at 4x magnification. 20 instruments of Group A (10 per system) were remained unused. 20 instruments of Group B (10 per system) were instrumented with 20 root canals of single-rooted mandibular premolars, each for 2 minutes (each file used once). 20 instruments of Group C (10 per system) were instrumented with 40 root canals of single-rooted mandibular premolars, each for 2 minutes (each file used twice). Last, 20 instruments of Group D (10 per system) were instrumented with 60 canals of single-rooted mandibular premolars, each for 2 minutes (each file used 3 times). These instruments underwent cyclic fatigue testing and were compared to new, unused instruments.

For standardizing the root canal instrumentation, the water pipes were used to hold the teeth, water pipes were cut to 25 mm in length and 25 mm in width, and used as a custom-made mold that held the samples with the help of addition silicon impression material (proclinic). Access cavity opened and the chamber filled with sodium hypochlorite, 10 K-file from (Dentsply Sirona) was used to establish the working length. A crown-down technique used to prepare the root canal; first, the orifice opener (tip 17, taper 0.12) (Fanta Dental, Shanghai, China) was used with in- and out-brushing movement, and then the canal orifice was filled with 10 ml of 2.5% NaOCl.

Root canal instrumentation:

a. Instrumentation by AF F-One (F5).

A total of 30 new files (AF F-ONE) of (tip 0.25, 0.06 taper) were selected and used with a speed of 500 RPM/2.8 N torque, under FWD-Clockwise continuous rotation mode using the eighteeth endomotor, 10 new files (B2) instrumented 10 premolar canals, each for 2 minutes. Other 10 new files (C2) instrumented 20 canals (each file prepared 2 canals, each with 2 minutes). Last, 10 new files (D2) instrumented 30 canals (each file prepared 3 canals, each with 2 minutes).

(b) Instrumentation by 2Shape (TS2).

A total of 30 new files size TS2 (tip 0.25, 0.06 taper) were selected and used with a speed of 300 RPM/2.5 N, under FWD-Clockwise continuous rotation mode using the eighteeth endomotor: 10 new files (B1) instrumented 10 premolar canals, for 2 minutes. Other 10 new files (C1) instrumented 20 canals (each file prepared 2 canals, each with 2 minutes). Last, 10 new files (D1) instrumented 30 canals (each file prepared 3 canals, each with 2 minutes).

In both systems, all root canals were instrumented in pecking motion until the instruments reached the apex, and during instrumentation, after every 3 in and out pecking motion, the file was cleaned by a gauze that was socked in alcohol, after every 1 minute. For instrumentation, 10 ml of NaOCl was used to irrigate the canal for all groups, and after each use, the files were ultrasonically cleaned in ethanol for 5 minutes and sterilized at 121°C at a 30 psi pressure for 20 minutes and dried for 15 minutes. Then, all the files were exposed to cyclic fatigue testing.

### 2.1. Cyclic Fatigue Test

A 1.5-mm-inner-diameter stainless steel artificial canal with a curvature radius of 5 mm and 50 degree angle curvature was used to assess and measure the CFR of all instruments (new and used). The working length of the artificial canal was fixed as 21 mm.

The software program was AutoCAD 2021 version used to draw the canal (see Figure 1), then transferred to form a frame of a pantograph that was analyzed by a hyper spark laser machine to make an artificial stainless steel canal.

The E-connect endomotor hand piece was connected to a dental surveyor for standardization purpose (see Figure 2), and then the instrument was fixed to the hand piece and placed in the canal, and the motor was run for each system according to manufacturer instructions until the instrument fractured (see Figure 3). To reduce excessive heating during rotation and to minimize the friction, the canal was lubricated. A digital camera (Canon d7500) was used to record a video of each instrument rotation until fracture, the time to fracture registered in seconds and then converted into the number of cycles to failure (NCF) by using the subsequent formula: rpm × time to failure in seconds/60.

Data were analyzed using SPSS 25 software (IBM-SPSS Inc, Chicago, IL, USA) for statistical analysis. The Welch ANOVA and Kruskal nonparametric method for evaluating the level of significance among instruments, the pairwise test for multiple comparisons, and the Mann–Whitney *U* test for inter-group comparison was used, with a level of significance at (*P* < 0.05).

## 3. Results

Table 1 shows the mean and standard deviation (SD) of the CFR of new and used instruments.

### 3.1. Within-Group Statistical Analysis

To identify the presence of significant differences between new instruments and used ones, since the data were scale-based, it was essential to test normality. Based on the below results (see Table 2), we confirmed that the datasets from the AF F-One group were normally distributed. The ANOVA test was used. Homogeneity assumption was taken into consideration and failed to accept the null hypothesis of equal variance due to small *P* values (0.007) < 0.05 as seen in Table 2. Therefore, the Welch test of comparison was performed, and there was a significant difference between the four applications of Fanta instruments.

For intragroup comparison, the pairwise multiple comparison test was used for the AF F-One group (see Table 3) and showed a significant decrease in the CFR in AF-F-One files after clinical use (*P* < 0.05), only the difference between files with two uses and files with three uses was not significant (*P* = 0.89).

With respect to the 2Shape/TS2 group, due to violating normality (see Table 4), where *P* values of all files were below 0.05. Thus, the Kruskal non-parametric method was used and according to its *P* value, no statistically significant differences were found between the instruments.

### 3.2. Between Groups Comparison

Statistical tests (Mann–Whitney *U*) showed a significant difference between (AF F-One and 2Shape groups) in all 4 applications (see Table 5).

## 4. Discussion

Fractured rotary NiTi instruments may fail due to cyclic flexural fatigue or torsional failure, or a combination of both (5). In this study, a method was used to estimate cyclic fatigue which has already been identified and used in several articles [9, 17–19].

The 2Shape TS2 (MicroMega, Besancon, France) and AF F-ONE (Fanta Dental Material Co., Shanghai, China) rotary instruments used in this study had the same #25 tip size and a constant 6% taper. The difference is the presence of a flat side design with an S-shaped cross-section in the F-One file and the fact that the file is made of AF-R wire. While the 2Shape features the latest cross-section generation with a triple helix with dual cutting edges for cutting efficiency and one secondary edge for better canal debridement, T-wire technology claims to increase the CFR by 40% when compared to One Shape (MicroMega) instrument [13, 14].

In the present study, a reduction in CFR was exhibited after the clinical use of AF F-One instruments. These results were expected because while shaping curved root canals at the maximum canal curvature continuous tensile and compressive stresses occur on NiTi rotary instruments that lead to fracture because of flexural fatigue [20]. In addition, the Fanta instruments have S-shaped cross-section, and the mean stress point and the speed of rotation in AF F-One (500 rpm) play another role; this is because the surface temperature of the file rises as the number of revolutions increases. [14, 21]

The study also found that clinical use did not affect the CFR of the 2Shape instrument (*P* > 0.05). Therefore, the initially tested null hypothesis was partially accepted.

T-Wire heat treatment used in 2Shape files construction can be a cause of the improved file's elasticity. This may be the reason for the higher fracture resistance of the 2Shape files after use when compared to the AF F-One files [22]. The CFR of endodontic instruments may be affected by not only the alloy characteristics but also by various factors [6, 23]. The rotational speed at which the instrument is used might affect the CFR because as the rotation speed increases, the surface temperature of the instrument increases, creating thermomechanical stress on the instrument and lowering the CFR [24].

This result is in agreement with a previously published study that compared the CFR of EndoSequence Xpress (ESX), 2Shape, Twisted File (TF), and NiTi rotary files. All instruments were rotated in an artificial canal made of stainless steel with a 1.5-mm inner diameter, radius curvature of 5 mm, and 60° curvature angle until a fracture occurred, NCF values showed that the 2Shape instruments had the highest CFR significantly [22].

The second result was that the mean NCF of AF F-One instruments was significantly higher than the equivalent file size of 2Shape instruments. Therefore, the second null hypothesis was not accepted. The reason behind this is considered due to AF F-One file being made of AF-R wire which is a developed NiTi alloy with more flexibility, good shape memory, and excellent mechanical properties. Moreover, a flat design has benefits in reducing torsional stresses by sweeping the debris from flutes to the relieving area, due to the smaller contact surface and the lower friction that produced when the file progresses into the canal [7, 25]. Since during rotation of the file inside the artificial canal less engagement of the file as well as friction occurs, the cyclic fatigue study could also be affected by this [25].

It is important to emphasize that the cost can be decreased with repeated use of the instruments. In contrast, as the number of uses increases, the chance of instrument fracture and the average time required for the instrumentation of the canal will increase, as the file will experience reduced surface roughness, fatigue, and cutting efficiency, as confirmed by other studies as well [26, 27].

The CFR of AF F-One files was affected adversely by the number of clinical uses. To evaluate how many times a rotary NiTi endodontic instrument could be used in root canals safely, more research studies are needed and to analyze it with other various rotary systems according to various aspects. Moreover, future studies are required to examine the clinical performance and evaluate other properties of these files to provide the clinician with valid and more conclusive information. It is also important to discard the instruments on a regular basis and not to surpass the maximum number of usage recommended by the manufacturer.

## 5. Conclusion

Within the limitations of the current study, a reduction in the CFR of AF F-One instruments was observed after clinical usage when compared to new groups. While the 2Shape system was not affected by clinical use. Furthermore, Fanta files had higher NCF than 2Shape ones and performed better.

## Figures and Tables

**Figure 1:** Dimensions of the artificial canal performed by (AutoCAD).

**Figure 2:** Dental handpiece fixation on the dental surveyor.

**Figure 3:** Instrument fracture.

**Table 1:** Descriptive statistics analysis of both groups.

Groups	Usage time	*N*	Mean ± SD	95% confidence interval for mean	
				Lower bound	Upper bound
AF F-ONE	New	10	3758.650 ± 1074.677	2989.872	4527.428
	One use	10	1547.700 ± 640.416	1089.574	2005.826
	Two use	10	1653.050 ± 360.143	1395.419	1910.681
	Three use	10	1754.900 ± 293.125	1545.211	1964.589
2Shape	New	10	766.200 ± 119.509	680.708	851.692
	One use	10	714.300 ± 81.147	656.251	772.349
	Two use	10	700.200 ± 89.924	635.872	764.528
	Three use	10	648.900 ± 135.934	551.659	746.141

**Table 2:** Normality, homogeneity, and ANOVA test outcome for instruments in AF F-one group.

Groups	Instrument type	Shapiro–Wilk (*P* value)	Homogeneity test	ANOVA test
			(*P* value)	(*P* value)
AF F-one	New	0.852 (0.062)	4.783 (0.007)	25.086 (0.000)
	One use	0.782 (0.065)		
	Two use	0.948 (0.645)		
	Three use	0.920 (0.358)		

**Table 3:** Pairwise multiple comparison result for AF F-one group.

AF F-one group		Mean difference (I–J)	Sig.	95% confidence interval	
				Lower bound	Upper bound
New	One use	2210.950^*^	0.000	1982.838	4105.862
	Two use	2105.600^*^	0.001	1026.864	3184.336
	Three use	2003.750^*^	0.001	932.312	3075.188
One use	Two use	−105.750^*^	0.000	−1296.485	−581.015
	Three use	−207.600^*^	0.000	−1332.950	−748.250
Two use	Three use	−101.850^*^	0.898	−518.540	314.840

∗= mean difference of number of cycles to fracture between two group of instruments.

- = number of cycles to fracture in this group was increased.

**Table 4:** Normality, homogeneity and Kruskal–Wallis test for 2Shape/TS2 group.

Groups	Instrument type	Shapiro–Wilk	Homogeneity test	Kruskal–Wallis
			(*P* value)	(*P* value)
2Shape/TS2	New	0.766 (0.006)	0.879 (0.461)	6.526 (0.089)
	One use	0.854 (0.065)		
	Two use	0.753 (0.004)		
	Three use	0.928 (0.429)		

**Table 5:** Between groups non-parametric pairwise comparison results.

Pairwise comparison	Mean difference	Mean rank difference	Mann–Whitney *U* (*P* value)
New/AF F-one–New/2Shape/TS2	2992.450	10.000	0.000 (0.000)
One use/AF F-one–one use/2Shape/TS2	833.400	9.200	4.000 (0.001)
Two use/AF F-one–two use/2Shape/TS2	952.850	10.000	0.000 (0.000)
Three use/AF F-one–three use/2Shape/TS2	1106.000	10.000	0.000 (0.000)

## Data Availability

The findings of this study are supported by data that are available upon request from the corresponding author.
